# Antidiarrheal Effect of 80% Methanol Extract and Fractions of the Leaves of *Ocimum lamiifolium* in Swiss Albino Mice

**DOI:** 10.1155/2022/6838295

**Published:** 2022-05-26

**Authors:** Muluken Adela Alemu, Yared Andargie, Weretaw Sisay, Teklie Mengie, Getaye Tessema Desta, Tewodros Ayalew Tessema, Rahel Belete Abebe, Eshetie Melese Birru, Sisay Tarekegn Gebyaw, Meaza Adugna Ayanaw

**Affiliations:** ^1^Department of Pharmacy, College of Medicine and Health Sciences, Debre Tabor University, Debre Tabor, Ethiopia; ^2^Department of Pharmacology, School of Pharmacy, College of Medicine and Health Sciences, University of Gondar, Gondar, Ethiopia; ^3^Department of Pharmacy, Tseda Health Science College, Gondar, Ethiopia

## Abstract

**Introduction:**

Worldwide, in children of under five years of age, diarrhea is responsible for more than 760,000 annual deaths. It is treated with both modern drugs and traditional medicinal plants, including *O. lamiifolium*. But the use of this plant as an antidiarrheal agent is not scientifically validated. Therefore, this study was aimed to evaluate antidiarrheal efficacy of the plant.

**Method:**

The leaf powder was macerated by 80% methanol and then fractionated using *n*-hexane, *n*-butanol, and distilled water. Antidiarrheal activity was evaluated through different models (castor oil-induced diarrhea, enteropooling, and motility) using onset, number of wet feces, fluid content, weight and volume of intestinal content, and motility as test parameters by administering treatment doses to groups of mice. Group I received 10 mL/kg of the dissolving vehicle, Group II received either loperamide or atropine, and Groups III-V received extract doses of 100, 200, and 400 mg/kg, respectively. One-way ANOVA was used to analyze the data, followed by Tukey's post-hoc test.

**Results:**

The crude extract exhibited a significant effect on the fluid content of feces at all tested doses. Additionally, the *n*-butanol and distilled water fractions revealed significant effects on onset of diarrhea at 400 mg/kg (*p* < 0.05), while the *n*-hexane fraction showed significant effects on number of wet feces, onset, and fluid content of feces at all tried doses. The crude extract and all the fractions (at 200 and 400 mg/kg) decreased the weight and volume of intestinal content significantly. Similarly, both the crude extract and distilled water fraction at 400 mg/kg as well as *n*-butanol and *n*-hexane fractions at 200 and 400 mg/kg showed meaningful differences on peristaltic index as compared to the negative control.

**Conclusion:**

The results revealed that the leaf extract of *O. lamiifolium* has an antidiarrheal activity, which supports the traditional medical practice.

## 1. Introduction

Diarrhea is a symptom characterized by the presence of watery or loose feces, occurring three or more times per day with increased frequency and decreased consistency [1]. It is the second leading cause of child morbidity and mortality in developing countries. Globally, it is estimated that there are 2.5 billion episodes and 760,000 diarrheal deaths annually in children under five years of age, accounting for 9% of the estimated total annual child deaths [1–3]. A review in 2021 estimated that the prevalence of diarrhea was 15.3% among children under five in sub-Saharan Africa [4]. In Ethiopia, diarrheal disease is a big issue, and it is one of the top 15 countries in which nearly three-quarters of child deaths occur due to diarrhea [1]. It is the country's second principal cause of death among children under five [5]. Although studies are reporting a decline in morbidity and death as a result of diarrhea, there are concerns about a potential rebound in the future due to ever-increasing urbanization [6].

Infectious agents (bacteria, viruses, and parasites) and noninfectious agents (irritable bowel syndrome, coeliac disease, and malignancies) may cause acute or chronic diarrhea. Acute diarrhea is the passage of loose stools more than three times per day for less than 14 days, while persistent diarrhea lasts between 14 and 30 days and chronic diarrhea persists for more than a month. Lack of hygiene, poverty, malnutrition, lack of good drinking water, and maternal education are the risk factors [2, 7].

Diarrhea may cause different complications like dehydration, hydroelectrolytic disorders, increased acidosis, and nutritional deficits/malnutrition, providing a strong basis for its appropriate management [8, 9]. Despite the fact that modern drugs are used in the treatment, many are associated with resistance and side effects such as QT interval prolongation, drug-drug interactions, and contraindications [10, 11], which justifies the search for new drugs. In addition, different parts of plants are used for the treatment of diarrhea. *Rhamnus cathartica, Cornus mas, Solanum hastifolium, Ecballium elaterium, Balanites rotundifolia, Amaranthus caudatus, Mentha longifolia, Berberis crataegina* [12], and *Ocimum lamiifolium* Hochst. ex. Benth [13, 14] are among some.

The leaf of *O. lamiifolium* (in Amharic called Damakessie) is customarily used for the treatment of diarrhea, stomach disorders, and abdominal pains [13–16], headache and febrile illness [17], cough [18], malaise [19, 20], and soreness [20]. It is also used for the treatment of cold, measles, eye infections [21], and used as mosquito repellent [16, 22]. Additionally, *in vivo* and *in vitro* studies with positive results were obtained for antimalarial, insecticidal, analgesic, anti-inflammatory, hepatoprotective, antipyretic, and antioxidant activities [23–29]. Furthermore, the methanol extract of the leaf of the plant was safe at 2000 mg/kg in Swiss albino mice [24].

The presence of chemical compounds including alkaloids, sterols, carbohydrates, glycosides, tannins, flavonoids, bornyl acetate, *p*-cymene, camphene, *a*-pinene, and sabinene was also reported from the essential oil analysis of *O. lamiifolium* [29–32]. These chemical components have antimicrobial, antibacterial, and antifungal properties [16, 25]. The leaf extract of the plant showed a broader spectrum of activity against the growth of *S. epidermidis, B. cereus, E. faecalis, L. monocytogenes, C. albicans, S. aureus, C. perfringens,* and *S. pyogenes* strains with MICs ranging from 64 to 512 mg/mL [33, 34].

As indicated in ethnobotanical studies, *O. lamiifolium* is used as an antidiarrheal agent in Ethiopia [13–16]. But it may be ineffective, toxic, and may have drug interactions [35, 36], which rationalizes this study for an efficacy test. Furthermore, the findings of this study may be used as the input for future research in this field.

## 2. Materials and Methods

### 2.1. Drugs and Chemicals

Drugs, chemicals, and reagents used in this study were of the required quality and were purchased from local suppliers. Distilled water (University of Gondar teaching specialized hospital, Ethiopia), methanol (Blulux, India), *n*-butanol (Blulux Laboratories Ltd, India), loperamide hydrochloride (Medochemie Ltd, Limassol Cyprus), castor oil (Amman Pharmaceutical Industries, Jordan), *n*-hexane (Pentokey organy, India), activated charcoal (Acuro Organics Ltd, New Delhi), Tween 80 (Atlas Chemical Industries Inc, India), atropine sulfate injection (JeilPharm. Co. Ltd., Korea), ferric chloride (Bdhltd, England), potassium ferrocyanide (BDH Ltd, England), Mayer's and Dragendorff's reagents (May and Baker Ltd, Dagenham, England), ammonia (Merck Millipore, India), lead acetate test (Fisher Scientific, UK), acetic anhydride (Techno Pharmchem, India), and sulfuric acid (Farm Italia Carlo Erba, Italy) were used in the experiment.

### 2.2. Plant Material

A sufficient amount of the leaf of *O. lamiifolium* was collected around Gondar city, Northwest Ethiopia, in August 2021. The use of the leaf of the plant in the present study complies with the IUCN (International Union for Conservation of Nature) Policy Statement on Research Involving Species which are endangered and at risk of extinction. A botanist from Gondar University's Biology Department authenticated the plant, and the specimen was deposited in the herbarium with voucher number (MA1). The normal fresh leaves of *O. lamiifolium* were first washed with clean water and then dried under shade. The dried leaves were crushed to a coarse powder.

### 2.3. Extraction and Fractionation

#### 2.3.1. Preparation of 80% Methanol Crude Extract

Extraction was conducted based on the method used by Chalalai et al. [37]. The powdered leaves (1.2 kg) were mixed with 80% methanol in 1 : 5 a ratio. The powder was macerated for 72 h at room temperature with repeated shaking and then filtered using a muslin cloth followed by a filter paper (Whatman No. 1). The marc was re-extracted two times by adding a similar volume of fresh 80% methanol. The filtered fluid extracts were poured into a container and evaporated to dryness at 40°C and then lyophilized. Then, the crude extract was stored in a refrigerator at 4°C until use.

#### 2.3.2. Fractionation

The methanolic crude extract was fractionated using distilled water, *n*-butanol, and *n*-hexane as fractionating solvents. The crude extract (100 g) was suspended in 350 mL of distilled water and was poured into a separatory funnel, and then the same volume of *n*-hexane was used to separate nonpolar phytochemicals. The mixture exhibited two layers, with the *n*-hexane layer being on top. The water part was collected in another beaker and fresh *n*-hexane was added again. Overall, *n*-hexane-based extraction was carried out three times separately. All the *n*-hexane filtrates were collected in one beaker and allowed to be dried in an oven at 40°C. On the remnant (aqueous layer), another 350 mL of *n*-butanol was added and shaken. Again, the aqueous layer was at the bottom. The *n*-butanol filtrate was collected in a beaker. Another 350 mL of *n*-butanol was added two more times separately to get the *n*-butanol fraction. The final remaining residue was an aqueous fraction. All the *n*-butanol extracts were collected in one beaker and then dried in an oven at 40°C while the aqueous residue was dried in a lyophilizer. All dried extracts were kept in an airtight container in the refrigerator until use.

### 2.4. Experimental Animals

An inbred either sex Swiss albino mice with an age range of 8–12 weeks and a weight range of 20–30 g were chosen (obtained from colonies in the animal unit of Department of Pharmacology, College of Medicine and Health Sciences, University of Gondar). They were housed in plastic cages with wood chip bedding and allowed free to water and food. They were kept in a room having light similar to the natural cycle (12 h on and 12 h off). Animals were allowed to adapt in the laboratory for 7 days before to the beginning of the experiment. Care and management of mice were performed according to OECD guideline 420 [38].

### 2.5. Animal Grouping and Dosing

For each of the solvent extracts and for each model, mice (*n* = 30) were randomly assigned from Group I to Group V (six animals per group). Group I was assigned as a negative control (took 10 mL/kg distilled water for methanol, aqueous, and *n*-butanol extracts as well as 10 mL/kg 2% tween-80 for *n*-hexane extract). Mice of group II (positive control) were given loperamide 3 mg/kg for two diarrhea models (castor oil-induced and enteropooling) while atropine sulfate 1 mg/kg was given in the motility model. Animals in Groups III to V were given 100, 200, and 400 mg/kg doses of the crude extract, *n*-butanol, water, and *n*-hexane fractions.

### 2.6. Phytochemical Screening of Leaves of *O. lamiifolium*

The presence or absence of flavonoids, anthraquinones, tannins, glycosides, saponins, terpenoids, phenols, alkaloids, and steroids was assessed for all extracts using standard evaluation methods [39].

### 2.7. Antidiarrheal Activity Determination

#### 2.7.1. Castor Oil-Induced Diarrhea

This model was conducted as described by Muluken et al [40]. For each extract, either sex of mice (*n* = 30) were randomly allocated to five groups and fasted food (pellet) but not water for 18 h. Dosing of extracts was performed as indicated in the grouping and dosing section. One h after dosing, castor oil (0.5 mL) was given orally, and then the mice were placed in a metabolic cage in which the floor was covered with a nonwetting transparent paper. The paper was changed every hour, and the mice were observed for four hours. During the experimental observation period (4 h), onset time of diarrheal stool, number of total stools, number of diarrheal stools, and weight of feces were recorded. Onset time was measured from the time of castor oil administration to the occurrence of the first diarrheal stool. Measurement parameters in the negative control group were taken as 100% to be used as a benchmark for the effect of extracts. Inhibition of diarrhea and defecation (percentage) were calculated using the following formula [41]:

(1) $$\begin{array}{c} \text{\%Inhibition of Diarrhea}=\frac{\text{Mean number of wet stools of}\left(\text{control group}-\text{treated group}\right)}{\text{Mean number of wet stools of control group}}\times 100, \end{array}$$

(2) $$\begin{array}{c} \text{\%Inhibition of defecation}=\frac{\text{Total number of feces in the }\left(\text{negative control}-\text{treated group}\right)}{\text{Total number of feces in the negative control}}\times 100. \end{array}$$

#### 2.7.2. Castor Oil-Induced Enteropooling

The method used by Chitme et al. [42] was followed to observe the effect of the crude extract and fractions on intestinal fluid accumulation. This effect was found through the measurement of weight and volume of small intestinal fluid. Thirty mice were grouped into five groups (six mice per group) and then fasted for both food and water for 18 h prior to administration of the extracts. Mice were dosed as described in the grouping and dosing section. One hour after dosing the extract, 0.5 mL of castor oil was administered orally. After about an hour, each mouse was sacrificed using the cervical dislocation method, and the small intestine was cut after tying the cecum and pyloric ends. Then, the weight of the intestine was measured. The volume of intestinal content was measured after expelling it into a graduated cylinder [42]. The empty intestine was reweighed again and the weight difference between the full and empty intestine was recorded. Percentage inhibition of weight and volume were calculated as follows:

(3) $$\begin{array}{c} \%\text{of inhibition by using MWIC}=\frac{\text{MWICC}-\text{MWICT}}{\text{MWICC}}\times 100, \end{array}$$

where MWIC—mean weight of intestinal content, MWICC—mean weight of intestinal content of the control group, and MWICT—mean weight of intestinal content of the test group. Moreover,

(4) $$\begin{array}{c} \%\text{of inhibition by using MVIC}=\frac{\text{MVICC}-\text{MVICT}}{\text{MVICC}}\times 100, \end{array}$$

where MVIC—mean volume of intestinal content, MVICC—mean volume of intestinal content of the control group, and MVICT—mean volume of intestinal content of the test group.

#### 2.7.3. Gastrointestinal Motility Test Model

Like in the abovementioned models, thirty mice were allocated to five groups and fasted food for 18 h. Then, the doses were given as explained in the grouping and dosing part. One hour after dosing, castor oil (0.5 mL) was given orally to each mouse. After oral gavage of castor oil, the mice were observed for 1 h and then 1 mL of charcoal meal (5% charcoal suspension in 2% tween-80) was given orally. One hour later, the mice were sacrificed using the cervical dislocation method, and then the small intestine was removed carefully by opening the abdomen in a way that could not affect the charcoal meal travel. The intestine was laid straight on a clean table. The charcoal travel length from the pylorus to the cecum was determined using a measuring ruler and showed as a percentage of the length of the whole small intestine [43].

(5) $$\begin{array}{c} \text{Peristalsis index}\left(PI\right)=\frac{\text{distance travelled by the charcoal meal}}{\text{total length of small intestine}}\times 100, \end{array}$$

(6) $$\begin{array}{c} \%\text{of inhibitio}=\frac{\text{PI of negative control}-\text{PI of drug or extract treated}}{\text{PI of negative control}}\times 100. \end{array}$$

The *in vivo* antidiarrheal indices (ADI) were computed using the formula formed by Than et al [44].

(7) $$\begin{array}{c} \text{ADI in vivo}=\sqrt[{3}]{\text{Dfreq}\times \text{Gmeq}\times \text{Pfreq}}, \end{array}$$

where *D* freq is the onset of diarrhea obtained from castor oil diarrhea model, calculated as follows:

(8) $$\begin{array}{c} \text{Dfreq}=\frac{\text{mean onset of diarrhea}\left(\text{in treated group}-\text{in the negative control group}\right)}{\text{mean onset of diarrhea in the negative control group}}\times 100. \end{array}$$

G meq is percent inhibition of motility, and P freq is percent inhibition of diarrhea.

### 2.8. Statistical Analysis

SPSS (version 26) was used to analyze the data and the results were expressed as a mean ± standard error of the mean (SEM). ANOVA (one-way analysis of variance) and then Tukey's multiple comparison test were used to identify the presence or absence of differences between groups. Differences between groups were considered meaningful if the *P*value was less than 0.05.

## 3. Results

### 3.1. Yields of the Plant

A total of 175 g of crude extract were obtained from the maceration of 1.2 kg of *O. lamiifolium* leaf powder (14.58% w/w). After fractionation of the crude extract by *n*-hexane, *n*-butanol, and distilled water, a total dried yield of 6.25 g (6.25% w/w), 20.5 g (20.5% w/w), and 73.25 g (73.25% w/w) were obtained, respectively.

### 3.2. Phytochemical Screening

As shown in Table 1, many phytochemical constituents were identified in the crude extract. Of these, the *n*-hexane fraction contained many kinds of phytochemicals; whereas, the distilled water fraction contained only a few kinds of phytochemicals.

### 3.3. Determination of Antidiarrheal Activity

#### 3.3.1. Castor Oil-Induced Diarrhea

In this model, the crude extract showed significant effect on onset time of diarrhea, number of diarrheal feces, and weight of fresh feces at 400 mg/kg dose (*p* < 0.05). Furthermore, the crude extract showed significant effect on fluid content of feces in contrast to the negative control (*p* < 0.001).

The distilled water and *n*-butanol fractions showed significant effect on onset of diarrhea at 400 mg/kg dose compared with the negative control (*p* < 0.05). In comparison with the negative control group, the *n*-hexane fraction revealed significant effects on onset time of diarrhea, total number of feces, number of diarrheal feces, and fluid content of feces at all tested doses. Similarly, the fraction showed significant effect on the weight of fresh feces at 400 mg/kg dose (*p* < 0.001) (Table 2).

#### 3.3.2. Effects on Castor Oil-Induced Enteropooling in Mice

At 200 and 400 mg/kg, the methanolic crude extract revealed a meaningful difference on the volume and weight of small intestinal content in contrast to the negative control. The distilled water, *n*-butanol, and *n*-hexane fractions showed significant effects (at 200 and 400 mg/kg) on both volume and weight of small intestinal contents (Table 3).

#### 3.3.3. Effects on Castor Oil-Induced Intestinal Transit in Mice

Both the crude extract and the distilled water fraction (400 mg/kg) showed significant effects on charcoal meal travel and peristaltic index parameters when correlated with the negative control. Similarly, the *n*-butanol fraction revealed significant effects on charcoal meal travel (400 mg/kg) and on peristaltic index (at doses of 200 and 400 mg/kg). Meaningful differences were observed on administration of the *n*-hexane fraction for both charcoal meal travel and peristaltic index parameters at 200 and 400 mg/kg doses when correlated with the negative control (Table 4).

### 3.4. Antidiarrheal Indices (ADI) Values

As shown in the Table (Table 5), the hexane fraction showed a greater ADI value compared to others. Based on ADI values, the crude extract and fractions were arranged in the increasing order as distilled water fraction < n-butanol fraction < crude extract < n-hexane fraction.

## 4. Discussion

The leaf of *O. lamiifolium* is customarily used for the treatment of diarrhea in Ethiopia [13–16]. However, antidiarrheal efficacy was not scientifically proven. So, the aim of this study was to validate the antidiarrheal efficacy of the leaf extract of *O. lamiifolium* using castor oil-induced diarrhea in mice.

The imbalance between absorptive and secretory processes in the gastrointestinal tract produces diarrhea. In experimental models, diarrhea is commonly induced by castor oil [40–42]. Ricinoleic acid, the active metabolite of castor oil, which is released upon the action of lipases in the small intestine, is a known agent to cause diarrhea [42, 43]. Ricinoleic acid causes the release of prostaglandins through intestinal irritation and inflammation mechanisms, which in turn increases intestinal motility as well as the secretion of water and electrolytes. The other mechanism to cause these effects is by activating G protein-coupled prostanoid receptor (EP3) on intestinal smooth muscle cells [45]. Additionally, it inhibits sodium-potassium ATPase by forming sodium and potassium ricinoleate salts in the lumen which may result in an increase in intestinal permeability [46].

In the castor oil-induced diarrhea model, the crude extract produced a significant antidiarrheal effect on many measured parameters like the onset of diarrhea, number of wet feces, and weight of fresh feces at 400 mg/kg (*p* < 0.05), while all tested doses of the crude extract had a meaningful difference on fluid content of feces (*p* < 0.001). The distilled water and *n*-butanol fractions at 400 mg/kg dose produced significant differences only on onset of diarrhea, while *n*-hexane fraction produced meaningful differences on all tested parameters. The high activity for *n*-hexane fraction in many parameters may be due to the presence of many secondary metabolites, including alkaloids, flavonoids, tannins, saponins, steroids, anthraquinones, and terpenoids. Anti-inflammatory agents like non-steroidal anti-inflammatory drugs (NSAIDs) prevent diarrhea through inhibition of prostaglandin synthesis. Similarly, the leaf extract of *O. lamiifolium* showed antioxidant activity [29]. Therefore, antidiarrheal activity of the extract of the leaf might be through inhibition of prostaglandin synthesis. Furthermore, the presence of phytochemicals like terpenoids and steroids may account for antidiarrheal activity because these phytochemicals are known to inhibit prostaglandin E synthesis, reducing intestinal secretion [47, 48]. Therefore, the observed higher activity of the *n*-hexane fraction may be due to the availability of these phytochemicals in the fraction.

The secretory component of diarrhea was assessed by the enteropooling model. The crude extract and all the fractions at doses of 200 and 400 mg/kg showed meaningful reductions in volume and weight of intestinal content as compared to the negative control. The increase in weight and volume of small intestinal content might be due to the activation of nitric oxide pathway through the effect of ricinoleic acid [49]. It is known that the presence of phytochemicals like flavonoids, terpenoids, alkaloids [50], and steroids [43] decreases the synthesis of nitric oxide. Tannins affect the activity cystic fibrosis transmembrane conductance regulator protein (a protein that transporters chloride ions from epithelial cells to the lumen) in a way that can reduce secretion in the small intestine and colon [51]. In addition, tannins reduce intestinal secretion by inhibiting intracellular Ca^2+^ inward current [52]. Furthermore, phenols are known to have antioxidant activity, which may involve in inhibition of inflammation [53].

In the third antidiarrheal activity assessment method (gastrointestinal motility model), the crude extract and distilled water fraction at 400 mg/kg (*p* < 0.01) dose, as well as the *n*-butanol and *n*-hexane fractions at 200 and 400 mg/kg doses revealed meaningful differences on peristaltic index as compared to the negative control. This antimotility activity may be due to the concerted effect of secondary metabolites. Flavonoids are known to inhibit intestinal motility [54]. Terpenoids also inhibit intestinal motility in the gut [55]. Studies revealed that tannins decrease peristaltic movements through inhibition of the intracellular Ca^2+^ inward current [52].

Antidiarrheal index (ADI) is used to evaluate antidiarrheal effect using different parameters from different models. It is a combined figure of D freq (delay in onset), G meq, (reduction of gut meal motility as % inhibition), and P freq (a decrease in the number of diarrheal stools as % inhibition). For all the extracts, the value increases with the dose. The higher ADI value for the *n*-hexane fraction indicates its superior antidiarrheal effect as compared to other extracts. The activity difference between the fractions may be due to differences in the attraction of phytochemicals both in quality and quantity to the fractionating solvents. As indicated in Table 1, *n*-hexane fraction was able to localize many phytochemical constituents which may be a reason for its superior activity.

## 5. Conclusion

This study revealed the methanolic crude extract and solvent fractions of the leaf of *O. lamiifolium* have antidiarrheal activity. Therefore, the findings of this study provide a scientific basis for the traditional use of the leaf of *O. lamiifolium* as an antidiarrheal agent in Ethiopian traditional medical practice.

## Figures and Tables

**Table 1:** Results of phytochemical screening for the extracts of *O. lamiifolium.*

Chemical constituents	80% Methanol extract	Fractions		
		*n*-Butanol	*n*-Hexane	Distilled water
Alkaloids	+	−	+	−
Flavonoids	+	+	+	+
Phenols	+	+	−	+
Tannins	+	+	+	−
Saponins	+	+	+	+
Steroids	+	+	+	−
Glycosides	+	−	−	+
Anthraquinones	+	+	+	−
Cardiac glycosides	−	−	−	−
Terpenoids	+	−	+	−

Key: (+) = present (−) = absent.

**Table 2:** Effects of the crude extract and fractions of the leaves of *O*. *lamiifolium* on castor oil-induced diarrhea model in mice.

Treatment	Onset of diarrhea (min)	Total no. of feces	Total no. of wet feces	Weight of fresh feces (*g*)	Fluid content of feces (*g*)	% Inhibition of weight	% Inhibition of defecation	% Inhibition of diarrhea
NC	57.00 ± 4.57	5.17 ± 0.87	3.67 ± 0.88	0.71 ± 0.93	0.55 ± 0.10	—	—	—
PC	148.33 ± 20.40^a3^	2.50 ± 0.43^a1^	1.17 ± 0.31^a1^	0.12 ± 0.02^a2^	0.03 ± 0.00^a3^	83.10	51.64	68.12
CE 100	77.83 ± 3.97^b3^	4.33 ± 0.56	2.83 ± 0.60	0.49 ± 0.10	0.17 ± 0.07^a3^	30.99	16.25	22.89
CE 200	84.67 ± 6.47^b2^	4.00 ± 0.52	2.33 ± 0.49	0.39 ± 0.07	0.14 ± 0.04^a3^	45.07	22.63	36.51
CE 400	107.67 ± 10.61^a1^	3.00 ± 0.26	1.33 ± 0.21^a1^	0.22 ± 0.04^a1^	0.07 ± 0.01^a3^	69.01	41.97	63.76
BF 100	73.67 ± 3.41^b3^	4.50 ± 0.43	3.17 ± 0.40	0.51 ± 0.09^b1^	0.27 ± 0.07	28.17	12.96	13.62
BF 200	79.50 ± 4.46^b3^	4.00 ± 0.45	2.83 ± 0.40	0.38 ± 0.05	0.21 ± 0.03	46.48	22.63	22.89
BF 400	108.33 ± 6.32^a1^	3.33 ± 0.49	2.00 ± 0.45	0.32 ± 0.07	0.19 ± 0.04	54.93	35.59	45.50
DF 100	69.17 ± 3.44^b3^	5.00 ± 0.26^b1^	3.33 ± 0.21^b1^	0.51 ± 0.09^b1^	0.29 ± 0.06^b1^	28.17	3.29	9.26
DF 200	75.17 ± 3.82^b3^	4.33 ± 0.42	3.00 ± 0.37	0.39 ± 0.06	0.24 ± 0.03	45.07	16.25	18.26
DF 400	103.83 ± 5.74^a1,b1^	3.50 ± 0.56	2.17 ± 0.48	0.34 ± 0.07	0.21 ± 0.03	52.11	32.30	40.87
NC^*∗*^	56.50 ± 3.52	5.00 ± 0.37	3.50 ± 0.43	0.68 ± 0.05	0.54 ± 0.05	—	—	—
PC^*∗*^	150.00 ± 5.09^a3^	2.17 ± 0.31^a3^	1.00 ± 0.26^a3^	0.10 ± 0.01^a3^	0.02 ± 0.00^a3^	85.29	56.60	71.43
HF 100	80.50 ± 4.24^a1,b3^	3.33 ± 0.42^a1^	2.00 ± 0.37^a1^	0.54 ± 0.07^b3^	0.24 ± 0.03^a3,b3^	20.59	33.40	42.86
HF 200	87.83 ± 3.19^a2,b3,e1^	2.83 ± 0.31^a2^	1.50 ± 0.22^a2^	0.47 ± 0.07^b2^	0.11 ± 0.01^a3,c1^	30.88	43.40	57.14
HF 400	112.33 ± 8.73^a3,b3,c2^	2.33 ± 0.21^a3^	1.33 ± 0.21^a3^	0.24 ± 0.06^a3,c2^	0.06 ± 0.01^a3,c2^	64.71	53.40	62.00

NC = negative control (dissolved in distilled water), PC = positive control (dissolved in distilled water), CE = crude extract, BF = *n*-butanol fraction, DF = distilled water fraction, NC^*∗*^ = negative control (dissolved in 2% tween-80), PC^*∗*^ = positive control (dissolved in tween-80), HF = *n*-hexane fraction,^a^ compared to negative control,^b^ compared to positive control,^c^ compared to 100,^d^ compared to 200,^e^ compared to 400,^1^*p* < 0.05,^2^*p* < 0.01,^3^*p* < 0.001.

**Table 3:** Effects of 80% methanol crude extract and solvent fractions of the leaves of *O. lamiifolium* on gastrointestinal fluid accumulation in mice.

Treatment	Volume of intestinal content (mL)	% Inhibition	Weight of intestinal content (*g*)	% Inhibition
NC	0.67 ± 0.11	—	0.75 ± 0.11	—
PC	0.21 ± 0.12^a3^	68.66	0.29 ± 0.03^a3^	61.33
CE 100	0.49 ± 0.05^b1^	26.87	0.55 ± 0.05	26.67
CE 200	0.31 ± 0.07^a2^	53.73	0.42 ± 0.08^a1^	44.00
CE 400	0.25 ± 0.03^a3^	62.69	0.33 ± 0.03^a2^	56.00
BF 100	0.51 ± 0.05^b1^	23.88	0.57 ± 0.05^b1^	24.00
BF 200	0.34 ± 0.07^a2^	49.25	0.45 ± 0.08^a1^	40.00
BF 400	0.28 ± 0.03^a2^	58.21	0.37 ± 0.02^a2^	50.67
DF 100	0.54 ± 0.05^b2^	19.40	0.59 ± 0.05^b1^	21.33
DF 200	0.36 ± 0.07^a1^	46.27	0.47 ± 0.08^a1^	37.33
DF 400	0.30 ± 0.03^a2^	55.22	0.39 ± 0.03^a2^	48.00
NC^*∗*^	0.63 ± 0.11	—	0.72 ± 0.11	—
PC^*∗*^	0.19 ± 0.02^a3^	69.84	0.25 ± 0.02^a3^	65.28
HF 100	0.45 ± 0.05	28.57	0.50 ± 0.05	30.56
HF 200	0.26 ± 0.07^a2^	58.73	0.36 ± 0.08^a2^	50.00
HF 400	0.22 ± 0.03^a2^	65.08	0.28 ± 0.03^a3^	61.11

NC = negative control (dissolved in distilled water), PC = positive control (dissolved in distilled water), CE = crude extract, BF = *n*-butanol fraction, DF = distilled water fraction, NC^*∗*^ = negative control (dissolved in 2% tween-80), PC^*∗*^ = positive control (dissolved in 2% tween-80), HF = *n*-hexane fraction,^a^ compared to negative control,^b^ compared to positive control,^c^ compared to 100,^d^ compared to 200,^e^ compared to 400,^1^*p* < 0.05,^2^*p* < 0.01,^3^*p* < 0.001.

**Table 4:** Effects of the crude extract and fractions of the leaves of *O. lamiifolium* on castor oil-induced gastrointestinal motility model in mice.

Treatment	Mean length of small intestine (cm)	Mean distance traveled by the charcoal meal (cm)	Peristaltic index (%)	% Inhibition
NC	49.50 ± 1.38	40.17 ± 1.58	81.05 ± 1.45	—
PC	52.00 ± 0.97	21.17 ± 1.99^a3^	40.79 ± 3.85^a3^	49.67
CE 100	51.00 ± 1.79	37.17 ± 1.82^b3^	73.28 ± 4.41^b3^	9.59
CE 200	49.17 ± 1.20	34.00 ± 2.54^b3^	68.82 ± 3.82^b3^	15.09
CE 400	48.17 ± 1.47	30.33 ± 0.84^a2,b1^	63.29 ± 2.62^a2b3^	21.91
BF 100	51.33 ± 1.28	35.67 ± 1.65^b3^	69.76 ± 3.90^b3^	13.93
BF 200	49.83 ± 1.51	33.83 ± 2.67^b3^	67.58 ± 3.82^a1,b3^	16.62
BF 400	50.83 ± 0.70	29.00 ± 0.73^a2,b1^	57.06 ± 1.31^a3,b2^	29.60
DF 100	49.00 ± 1.39	37.33 ± 1.73^b3^	76.57 ± 4.42^b3^	5.37
DF 200	50.33 ± 1.98	35.83 ± 2.61^b3^	71.70 ± 5.66^b3^	11.54
DF 400	50.67 ± 1.63	30.50 ± 0.85^a2,b2^	60.69 ± 3.20^a2,b1^	25.12
NC^*∗*^	50.67 ± 1.73	38.33 ± 1.48	75.76 ± 2.22	-----
PC^*∗*^	51.33 ± 1.26	19.33 ± 2.08^a3^	37.83 ± 4.22^a3^	50.07
HF 100	50.00 ± 1.57	34.17 ± 1.81^b3^	68.43 ± 3.50^b3^	9.68
HF 200	50.00 ± 1.65	30.50 ± 2.51^a1,b2^	60.76 ± 3.74^a1,b3^	19.80
HF 400	47.83 ± 1.89	25.83 ± 0.95^a3,c1^	54.37 ± 2.60^a2,b1,c1^	28.23

NC = negative control (dissolved in distilled water), PC = positive control (dissolved in distilled water), CE = crude extract, BF = *n*-butanol fraction, DF = distilled water fraction, NC^*∗*^ = negative control (dissolved in 2% tween-80), PC^*∗*^ = positive control (dissolved in 2% tween-80), HF = *n*-hexane fraction,^a^ compared to negative control,^b^ compared to positive control,^c^ compared to 100,^d^ compared to 200,^e^ compared to 400,^1^*p* < 0.05,^2^*p* < 0.01,^3^*p* < 0.001.

**Table 5:** *In vivo* antidiarrheal indices (ADI) of 80% methanol crude extract and fractions of the leaves of *O. lamiifolium*.

Treatment	D freq (from castor oil-induced diarrhea)	G meq (from charcoal meal test)	P Freq (from castor oil-induced diarrhea)	ADI
NC	—	—	—	—
PC	160.23	49.67	68.12	81.54
CE 100	36.54	9.59	22.89	20.02
CE 200	48.54	15.09	36.51	29.90
CE 400	88.89	21.91	63.76	49.89
BF 100	29.25	13.93	13.62	17.7
BF 200	39.47	16.62	22.89	24.67
BF 400	90.05	29.60	45.50	49.5
DF 100	21.35	5.37	9.26	10.20
DF 200	31.88	11.54	18.26	18.87
DF 400	82.16	25.12	40.87	43.86
NC^*∗*^	—	—	—	—
PC^*∗*^	165.49	50.07	71.43	83.96
HF 100	42.48	9.68	42.86	26.02
HF 200	55.45	19.80	57.14	39.73
HF 400	98.81	28.23	62.00	55.71

NC = negative control (dissolved in distilled water), PC = positive control (dissolved in distilled water), CE = crude extract, BF = *n*-butanol fraction, DF = distilled water fraction, NC^*∗*^ = negative control (dissolved in 2% tween-80), PC^*∗*^ = positive control (dissolved in 2% tween-80), HF = *n*-hexane fraction.

## Data Availability

The datasets are available from the corresponding author upon reasonable request.
